# Fractal Based Analysis of the Influence of Odorants on Heart Activity

This article has been retracted.

**DOI:** 10.1038/srep38555

**Published:** 2016-12-08

**Authors:** Hamidreza Namazi, Vladimir V. Kulish

**Affiliations:** 1 School of Mechanical and Aerospace Engineering, Nanyang Technological University, Singapore

## Abstract

An important challenge in heart research is to make the relation between the features of external stimuli and heart activity. Olfactory stimulation is an important type of stimulation that affects the heart activity, which is mapped on Electrocardiogram (ECG) signal. Yet, no one has discovered any relation between the structures of olfactory stimuli and the ECG signal. This study investigates the relation between the structures of heart rate and the olfactory stimulus (odorant). We show that the complexity of the heart rate is coupled with the molecular complexity of the odorant, where more structurally complex odorant causes less fractal heart rate. Also, odorant having higher entropy causes the heart rate having lower approximate entropy. The method discussed here can be applied and investigated in case of patients with heart diseases as the rehabilitation purpose.

Electrocardiography (ECG or EKG) is the process of recording the electrical activity of the heart over a period of time using electrodes placed on the skin. ECG has been used widely by scientists for monitoring heart activity. Besides analyzing the nature of ECG signal, many scientists have tried to analyze the influence of different kinds of external stimulation on heart activity. The works reported on analyzing the influence of auditory^1^,^2^,^3^, visual^4^,^5^,^6^ and olfactory stimuli^7^,^8^,^9^ are noteworthy to mention.

One useful method to study different types of biological signals is fractal method. A fractal is a natural phenomenon or a mathematical set that exhibits a repeating pattern displaying at every scale (self-similar). The scaling rules are characterized by “scaling exponents” (dimension). “Simple” regular fractals have integer scaling dimensions. Complex self-similar objects have non-integer dimension. Fractals can be defined as geometric objects whose scaling exponent (dimension) satisfies the Szpilrajn inequality^10^:



where  is the scaling exponent (dimension) of the object and *D*_*T*_ is its topological dimension, that is, Euclidean dimension of units from which the fractal object is built. In fact, Fractal and Euclidean geometries are conjugate approaches. Fractal geometry builds complex objects by applying simple processes to complex building blocks; Euclidean geometry uses simpler building blocks but frequently requires complex building processes^10^. Fractal time series shows the long-range correlations, meaning that each fluctuation in the time series is correlated with last fluctuations (memory concept), where the correlations change based on power law^11^. Fractal theory has been used widely in biology and medicine for various cases such as DNA^12^, eye movement^13^, EEG signal^14^, bone structure^15^, respiration signal^16^, human stride time series^17^ and face^18^.

In case of using fractal theory for analysis of ECG signals many works have been reported in literatures. D’Addio *et al*.^19^ performed fractal analysis on cardiac patients during resting, stress, early and late recovery phases of ECG stress test. They found out a significant change in fractal dimension values from resting to stress phase. In another work, Bhaduri and Ghosh^20^ did the fractal analysis on ECG signal of subjects performing Kundalini Yoga and Chi meditation. The result of their study showed enhancing complexity of the cardiac dynamics during meditation. Ghosh *et al*.^21^ used fractal analysis for comparison of ECG signal between healthy subjects and subjects suffering from Intracardiac Atrial Fibrillation. The result of their analysis showed that fractal dimension in case of Intracardiac Atrial Fibrillation has significant higher values compared to the normal ECG signal. This result indicates increasing ECG complexity for Intracardiac Atrial Fibrillation. See also^22^,^23^,^24^.

On the other hand, some researchers have focused on analyzing the entropy of ECG signal. They have employed different types of entropy for this purpose. For instance Kamath^25^ examined Renyi and Shannon entropy for discriminating normal and Ventricular. tachycardia or fibrillation (VT-VF) subjects. He found out that Renyi entropy outperforms Shannon entropy for this purpose with very high sensitivity, specificity, predictively and accuracy. In another work, Joseph *et al*.^26^ analyzed the effect of reflexological stimulation on heart rate variability. The result of their study showed the increment of Kolmogorov–Sinai entropy in reflexological stimulation compare to relaxed sitting, which indicates that the ECG signal becomes more random with reflexology. Baumert *et al*.^27^ explored the influence of head-up tilt and mental arithmetic stress on beat-to-beat variability of heart rate and QT interval, by computing sample entropy and cross-sample entropy. Based on their founding, head-up tilt resulted in a significant reduction in sample entropy of R-R intervals and cross-sample entropy, while mental arithmetic stress resulted in a significant reduction in coupling directed from R-R to QT. See also^28^,^29^,^30^.

Besides all the efforts done on the analysis of ECG signal using fractal approach, no work has been reported that studies the influence of olfactory stimulus (odorant in this research) on fractal dynamics of ECG signal. In this research, we hypothesize that there should be a correlation between odorant’s molecular complexity and the ECG signal fractal dynamics. In another step, we analyze the correlation between entropy of odorant and ECG signal.

## Method

In order to investigate the effect of odorant’s complexity on fractality of heart rate, the odorant’s complexity should be quantified. For this purpose, we considered the molecular complexity of odorants. In general, bigger and/or less symmetric molecules have higher molecular complexity. The molecular complexity (*C*) of an odorant is defined using Bertz formula^31^:



In this equation, *C*_*n*_ and *C*_*e*_ are functions of bond connectivity (*n*) and element diversity or kinds of atoms respectively.

The fractal dimension can be determined using some methods that approximate scaling and detail from limits estimated from regression lines over log vs. log plots of size vs. scale. There are several formal mathematical definitions such as box counting, information dimension and correlation dimension for computation of fractal dimension^32^. All these methods can be seen as special cases of a continuous spectrum of generalized fractal dimensions. Here we define this generalized fractal dimension. The fractal exponent is based on the entropy concept for a probability distribution^33^. For instance in case of a time series with range of variation between V_max_ and V_min_, we can divide the total range into N bin, where each bin has the size of δ ∈ :



So, the probability of a value to fall into the i’th bin:



In Equation (4) N_i_ is the number of times the value falls into the i-*th* bin. For a time series, it can be written as:



In Equation (5), t_i_ stands for the total time that the value spends in the i-th bin, and T is the total time.

The generalized fractal dimensions of order q defined by^34^:



where ∈ is the scaling factor.

As another parameter to investigate, we study the influence of odorant’s entropy at 25 °C on the entropy of heart rate. As it is known, at 0 °K odorants have zero entropy and as the temperature increases, their entropy increases.

In order to investigate the influence of odorant’s complexity and entropy on fractality and entropy of heart rate, we selected five pleasant odorants (look at Table 1) from Fenaroli’s Handbook of Flavor Ingredients^35^.

As it is shown Table 1, the odorants have molecular complexities in the range of 55.4 (Benzyl alcohol) and 177 (Diethyl malate). The molecular structures of selected odorants are shown in Fig. 1. It was mentioned that in general, bigger and/or less symmetric molecules have higher molecular complexity.

Also, as it is shown in Table 1, the odorants have entropy in the range of 85.55 (Benzyl alcohol) to 145.50 (Diethyl malate). The values of odorants’ entropies in 25 °C were collected from (http://realtime.molinstincts.com/).

### Data collection

The experiments were conducted on forty healthy students (look at Table 2). A physician examined subjects before the experiment to ensure that subjects are healthy. Subjects did not drink beverages which contain alcohol/caffeine within 48 hours before the experiments.

We have explained the study to subjects and then collected the informed consent from them. The Internal Review Board of Nanyang Technological University approved all procedures (including experimentation on human subjects), and we did our study based on the approved guidelines.

As un-wanted external stimuli can affect the data recording, we did the experiments in an isolated room from external stimuli. Subjects were lying down on the bed comfortably (supine position) during the data collection and instructed to focus on their breathing without doing any other job.

In order to find out the most effective concentration for each odorant, we did the preliminary experiments which analyze the effect of changing of odorants’ concentrations (by dilution) on the fractal dimension and approximate entropy of heart rate. We found out that odorant concentration in the range of “detection threshold” did not cause any significant change in heart rate, but odorant concentration over “recognition threshold” affected the heart rate. We found the most effective concentration for each odorant by considering the pleasantness level of odorant sensed by subjects, the allowable level that heart rate can be increased/decreased in the experiments and also task difficulty. The selected odorants showed the similar level for the most effective concentration. So, for our main experiments, we diluted odorants in mineral oil in order to equalize their concentrations in the observed most effective level and achieved an approximate gas-phase partial pressure of 1 Pa. We also measured the concentrations of odorants using an olfactometer which was connected to a gas analyzer, to ensure that the resulting vapor concentrations did not differ. The presentation of each odorant to gas analyzer was done 5 times (each time for 3 seconds) with inter-stimulus interval of 2 minutes.

We have noninvasively recorded ECG signal (cardioscope Oli Monitor 432, Kone Instrument Division) from the left middle finger, and analog-to-digitally converted with a sampling rate of 200 Hz. Data acquisition was initiated 15 min after the start of experiment to have stabilized hemodynamics. During measurement, the breathing of subjects was paced (breathing rate was 0.25 Hz) with a sound signal.

At first, the data collection was done free of any stimulus. Then, we presented different odorants in separate experiments to the subject’ nose using a 10 ml vial, and subject sniffed the odorants, and we recorded the ECG signal for 3 minutes. It is noteworthy we considered inter-stimulus time of 15 minutes between different odorants’ presentations.

In the second day, we repeated the data collection where in total two trials were collected from each subject for each stimulus. A physician controlled all experiments.

### Data analysis

After data collection, the physician checked all recorded heart rate data to ensure they are normal. All data were normal. So, we didn’t exclude any recorded data from analysis. Since the recorded ECG signal is noisy, in order to find heart rate (expressed in terms of R-R interval time series) we needed to filter the ECG signal. For this purpose we wrote a set of codes to do filtering. The low-frequency cutoff (high-pass filter) was set at 0.05 and 0.5 Hz. Low-pass filters were set at 40, 100, and 150 Hz (high-frequency cutoff). After filtering of the signal, another algorithm detects QRS complex (look at Fig. 2) followed by interpolation of R peaks. The R-R intervals^36^ were detected with a temporal resolution of 2 ms and then the R-R interval time series was generated.

The generated R-R interval time series were processed for computing of fractal dimension and entropy using other code. The written code computed the fractal dimension and entropy of R-R interval time series based on Box counting method^37^ and approximate entropy techniques^38^ respectively. Approximate entropy is indicator of randomness of time series where lower value of approximate entropy stands for less randomness. It is noteworthy that size of 11 was chosen for boxes based on literatures^39^,^40^,^41^. Also, the embedded time delay of 1 was chosen. All of these analyses were done in MATLAB.

### Statistical analysis

Mean values of fractal exponent and approximate entropy for the R-R interval time series were compared between different conditions using one-way repeated measures ANOVA. Mauchly’s test (*α* = 0.05) was conducted to test the sphericity. In fact, Mauchly’s sphericity test is a statistical test used to validate a repeated measures analysis of variance (ANOVA). Trend analysis was conducted based on the odorants’ properties. Omega squared (*ω*^2^) was used for a repeated measures design. Effect size, *r* was employed for pairwise comparisons. The statistical analyses were performed using SPSS (ver. 16.0).

## Results

Mauchly’s test indicated that the assumption of sphericity had not been violated in case of outcomes (fractal exponent and approximate entropy of R-R interval time series). The variations of fractal dimension for R-R interval time series due to different odorants and the odorants’ molecular complexities are shown in Fig. 3. The results stand for the mean values.

Since *F*_*crit*_(5,234) = 2.25 at *α* = 0.05, the statistical analysis result [*F*(5,234) = 50, p = 0.001] stands for the significant influence of odorants on the fractal dimension of R-R interval time series, with the effect size *ω*^2^ = 0.48. Generally, the application of the odorant reduced the fractal dimension of R-R interval time series. Olfactory stimuli conditions had a significant linear trend (*p* = 0.007), which indicates that Diethyl malate caused a greater variation in the fractality of R-R interval time series than Diethyl succinate, followed by Diethyl malonate, Dimethyl succinate and Benzyl alcohol respectively, reflecting the trend of molecular complexity of the odorants. The effect sizes in Table 3 show that Diethyl malate caused the greatest change in the fractality of R-R interval time series.

The variations of approximate entropy for R-R interval time series due to different odorants and the odorants’ entropy are shown in Fig. 4. The results stand for the mean values.

Since *F*_*crit*_(5,234) = 2.25 at *α* = 0.05, the statistical analysis result [*F*(5,234) = 61.5, p = 0.001] stands for the significant influence of odorants on approximate entropy of R-R interval time series, with the effect size *ω*^2^ = 0.56. Generally, the application of the odorant reduced the approximate entropy of R-R interval time series. Olfactory stimuli conditions had a significant linear trend (*p* = 0.026), which indicates that Diethyl malate caused a greater variation in the approximate entropy of R-R interval time series than the Diethyl succinate, followed by the Diethyl malonate, Dimethyl succinate and Benzyl alcohol respectively, reflecting the trend of entropy of the odorants. The effect sizes in Table 3 show that Diethyl malate caused the greatest change in the approximate entropy of R-R interval time series.

In overall, the correlation between the characteristics of odorants and the ECG signal was observed, where the odorant having higher complexity and entropy causes the greater change in fractality and entropy of R-R interval time series.

## Conclusion and Discussion

In this research we studied the effect of odorant’s complexity and entropy on fractality and approximate entropy of heart rate. Our results demonstrated the relation between heart rate and olfactory stimulus (odorant in this research), as the trend of the complexity of odorants is reflected on the trend of the reduction of fractality of R-R interval time series. For instance, Diethyl malate with highest value of molecular complexity caused greatest variation in fractality of R-R interval time series, compared to other odorants. This behaviour was seen in comparison between other odorants as well. On the other hand, the result of our analysis showed the similar trend of variations in case of odorant’s entropy and the approximate entropy of R-R interval time series. In overall, the correlation between characteristics of odorant and heart rate was observed, where the odorant having higher complexity and entropy causes the greater change in fractality and entropy of heart rate.

In fact, our study showed that beside the variation of heart rate due to olfactory stimulation, the characteristics of heart rate and olfactory stimulus are related. It means that our investigation is one step forward compared to studies that just investigated the influence of odorants on heart rate variability. In this way, the works which investigated heart rate variability due to olfactory stimulation using lemon and rose aromas^42^, sweet fennel oil^43^, sweet orange aroma^44^ and lavender^45^ are noteworthy to mention.

The behavior seen in this research can be explained through heart-brain connection. As it is known, heart activity is controlled by the nervous system where the brain is on its top. When human smells an odorant, olfactory neurons (as receptor cells) detect odor molecules and transmit information about the odor to the brain in a process called sensory transduction which yields to perception^46^. Based on the research done by Kermen *et al*.^47^, high complexity odorants activate more types of olfactory receptor than low complexity odorants. Thus, accordingly more information will be sent to the brain. Then, they will have stronger effect on the brain. Also, in ref. 48 we showed that complexity and entropy of the EEG signal (as a feature of brain activity) is coupled with the molecular complexity and entropy of the odorant, where more structurally complex odorants have greater effect on the EEG signal. On the other hand, based on the founding of scientists about the correlation between heart and brain through complexity analysis of EEG and ECG^49^,^50^, we hypothesize that the stronger effect on human brain which was caused by a more complex odorant, will shows its greater effect on the ECG signal, which is mapped on greater variation of its fractal dimension and entropy. This hypothesis needs to be worked on more by simultaneous analysis of the effects of different odorants with different molecular complexities on human EEG and ECG signals.

In this research, we did our analysis on healthy subjects. Several scientists have analyzed the effect of external stimulation on the heart rate of patients with different heart diseases. The works on analysis of the influence of lavender^51^,^52^, and the blend of oils of lemon, lavender, and ylang ylang^53^ as aromas on heart rate variability of patients are noteworthy to mention. In further attempts, our method also may be investigated in analysis of the influence of odorants on the heart rate of patients suffering from different heart diseases, where the diseases affect their heart rate. If our method works well in that case, we can continue our attempts with the rehabilitation purpose. Also, in further investigation, the method used in this research can be investigate in case of analysis of the influence of other kinds of external stimuli on heart activity.

Also, our analyses can help the current efforts for modeling of heart reaction to external stimulation. For instance, the result of our investigation in this research can be linked with our Fractional Diffusion Model of brain reaction to external stimulation in ref. 11, in order to write the observed correlation in the mathematical form.

## Additional Information

**How to cite this article**: Namazi, H. and Kulish, V. V. Fractal Based Analysis of the Influence of Odorants on Heart Activity. *Sci. Rep.* **6**, 38555; doi: 10.1038/srep38555 (2016).

**Publisher’s note:** Springer Nature remains neutral with regard to jurisdictional claims in published maps and institutional affiliations.

## Figures and Tables

**Figure 1:** Molecular structure of selected odorants.

**Figure 2:** A schematic of QRS complex.

**Figure 3:** Fractal dimension for R-R interval time series due to different odorants (left side), and the odorants’ molecular complexities (right side). Error bars indicate standard deviations.

**Figure 4:** Approximate entropy for R-R interval time series due to different odorants (left side), and the odorants’ entropies (right side). Error bars indicate standard deviations.

**Table 1:** Characteristics of odorants.

Name	Compound	Molecular complexity	Entropy
Benzyl alcohol	C7H8O	55.4	85.55
Dimethyl succinate	C6H10O4	114	118.24
Diethyl malonate	C7H12O4	125	132.42
Diethyl succinate	C8H14O4	135	136.29
Diethyl malate	C8H14O5	177	145.50

**Table 2:** Subjects characteristics.

Characteristic	Description
Sex	20 male and 20 females
Age	22.5 ± 0.5 years old
Height	172 ± 10.2 cm
Weight	71.5 ± 13.3 kg
Race	Indian
Ethnicity	Singaporean

**Table 3:** Effect sizes for pairwise comparisons.

Condition	Fractal dimension Effect size (r)	Approximate entropy Effect size (r)
No odorant vs. Benzyl alcohol	0.46	0.51
No odorant vs. Dimethyl succinate	0.74	0.75
No odorant vs. Diethyl malonate	0.82	0.84
No odorant vs. Diethyl succinate	0.83	0.85
No odorant vs. Diethyl malate	0.84	0.87
Benzyl alcohol vs. Dimethyl succinate	0.25	0.31
Benzyl alcohol vs. Diethyl malonate	0.38	0.55
Benzyl alcohol vs. Diethyl succinate	0.46	0.62
Benzyl alcohol vs. Diethyl malate	0.54	0.70
Dimethyl succinate vs. Diethyl malonate	0.20	0.35
Dimethyl succinate vs. Diethyl succinate	0.35	0.48
Dimethyl succinate vs. Diethyl malate	0.48	0.61
Diethyl malonate vs. Diethyl succinate	0.20	0.21
Diethyl malonate vs. Diethyl malate	0.39	0.40
Diethyl succinate vs. Diethyl malate	0.21	0.19
